# Mutation pattern is an influential factor on functional mutation rates in cancer

This article has been retracted.

**DOI:** 10.1186/s12935-016-0278-5

**Published:** 2016-02-09

**Authors:** Chuance Du, Xiaoyuan Wu, Jia Li

**Affiliations:** 1 Department of Urology, Ganzhou Hospital Affiliated to Nanchang University, Ganzhou, Jiangxi province China; 2 Department of Rehabilitation, Ganzhou Hospital Affiliated to Nanchang University, Nan Chang, Jiangxi province China; 3 Department of Thyroid and Breast, Shanghai Tenth People’s Hospital, Tongji University, Shanghai, 200072 China

**Keywords:** Clear-cell renal cell carcinoma, Liver cancer, Lung cancer, Melanoma, Mutation pattern, Random forest, Functional variants

## Abstract

**Background:**

Mutation rates are consistently varied in cancer genome and play an important role in tumorigenesis, however, little has been known about their function potential and impact on the distribution of functional mutations. In this study, we investigated genomic features which affect mutation pattern and the function importance of mutation pattern in cancer.

**Methods:**

Somatic mutations of clear-cell renal cell carcinoma, liver cancer, lung cancer and melanoma and single nucleotide polymorphisms (SNPs) were intersected with 54 distinct genomic features. Somatic mutation and SNP densities were then computed for each feature type. We constructed 2856 1-Mb windows, in which each row (1-Mb window) contains somatic mutation, SNP densities and 54 feature vectors. Correlation analyses were conducted between somatic mutation, SNP densities and each feature vector. We also built two random forest models, namely somatic mutation model (CSM) and SNP model to predict somatic mutation and SNP densities on a 1-Kb scale. The relation of CSM and SNP scores was further analyzed with the distributions of deleterious coding variants predicted by SIFT and Mutation Assessor, non-coding functional variants evaluated with FunSeq 2 and GWAVA and disease-causing variants from HGMD and ClinVar databases.

**Results:**

We observed a wide range of genomic features which affect local mutation rates, such as replication time, transcription levels, histone marks and regulatory elements. Repressive histone marks, replication time and promoter contributed most to the CSM models, while, recombination rate and chromatin organizations were most important for the SNP model. We showed low mutated regions preferentially have higher densities of deleterious coding mutations, higher average scores of non-coding variants, higher fraction of functional regions and higher enrichment of disease-causing variants as compared to high mutated regions.

**Conclusions:**

Somatic mutation densities vary largely across cancer genome, mutation frequency is a major indication of function and influence on the distribution of functional mutations in cancer.

**Electronic supplementary material:**

The online version of this article (doi:10.1186/s12935-016-0278-5) contains supplementary material, which is available to authorized users.

## Background

Cancer is a malignant disease as the result of the accumulation of somatic mutations (base pair substitutions, insertions, deletions, rearrangements and copy number changes) and the disruption of functions of critical genes and pathways in normal cells. Over the past 10 years, the rapid development and wide application of sequencing technology have enabled a full detection of somatic mutations in cancer genome. The big projects, such as The Cancer Genome Atlas and International Cancer Genome Consortium projects, have sequenced more than 25 thousand cancer genomes and exomes and provided tremendous mutation data, which facilitates a broad evaluation of mutation patterns and their roles in cancer initiation and development [1, 2]. Studies have consistently shown that somatic mutation rates are not constant across cancer genome and a variety of genomic properties influence local mutation densities, for instance, mutation frequency is increased close to breakpoints of structural rearrangements [3]. Mutagenesis is also highly affected by genomic features such as replication timing [4, 5], transcription levels [6] and chromatin organizations [7] in various cancer types.

It’s well accepted that somatic mutations play a pivotal role in carcinogenesis, however the extent to which mutation frequency affects cancer formation and development isn’t completely understood. For example, tumor cells with enhanced mutation frequency are prone to accumulation of driver mutations that confer a growth advantage to tumor cells and therefore are likely to develop cancer [8]. Hypermutated cancer genome possesses the prevalent signatures in genes which are critical to cancer initiation and progression [9, 10]. Moreover, recurrently mutated genes in a cohort of patients are regarded as cancer-driving genes under positive selection in cancers [6, 11]. However, few studies have been conducted on the function potential of mutation spectrum and its relation with functional somatic mutations in cancer. In this study, we characterized mutation patterns of four cancer types, including ccRCC, liver cancer, lung adenocarcinoma and melanoma. We observed a wide range of genomic features which affect local mutation rates and showed the importance of mutation frequency with respect to functionalities of somatic mutations. Low mutated regions have higher densities of deleterious mutations, higher average scores of non-coding variants, higher fraction of functional regions, and higher enrichment of disease-causing variants from HGMD and ClinVar databases than high mutated regions, supporting that mutation frequency is an important indicator of function and exerts a great impact on the distribution of functional mutations in cancer genome.

## Results

### The somatic mutation profile in cancer

To investigate the mutation pattern and what factors influence mutation rates in cancers, we obtained 71,424 somatic mutations from 14 paired ccRCC and normal samples [12], 2,011,261 variants from 25 melanoma patients [13], 1,845,976 from 24 lung adenocarcinoma patients, and 881,136 from 88 liver cancer patients [6] (see “Methods” section). We also took 38,248,779 SNPs (single nucleotide polymorphism) from the 1000 genomes project pilot one [14] as a comparison. We intersected somatic mutations and SNPs with a wide range of genomic features, epigenetic properties and computed the average mutation densities of somatic mutations and SNPs for each feature type. Figure 1 and Additional file 1: Figure S1–S4 showed the somatic mutation and SNP densities associated to various features. We found functionally important regions, such as CDS, promoter, UTR and ncExons are relatively low mutated compared to introns of lncRNAs (*P* value <0.05 in most cases except for promoter in kidney cancer and ncExon in melanoma and CDS, UTR for SNPs, Wilcoxon rank sum test). Furthermore, we obtained 5 cancer driver genes in ccRCC, VHL, PBRM1, TCEB1, BAP1 and SETD2, from Sato’s study [12], we found only two mutations, one in the CDS and another in the promoter of PBRM1, suggesting the CDS, promoters and UTR of these cancer-driving genes are mainly protected from mutations in ccRCC. Exons of either protein coding genes or lncRNAs showed lower somatic mutation rates relative to their introns respectively (*P* value <0.05 for lncRNAs in all cases, *P* value <0.05 for protein coding genes in liver and lung cancer, Wilcoxon rank sum test). However, no significant difference was observed on the SNP density between exons and introns of either protein coding genes or lncRNAs (*P* value >0.05 in all cases, Wilcoxon rank sum test). Expression level and replication time are two important factors affecting cancer mutation and SNP rates, as evidenced by consistently lower mutation and SNP rates in high expressed and early replicated genes versus low expressed and late replicated ones (*P* value <0.05 in all cases with a range from 0.008 to 2.429e-13, Wilcoxon rank sum test). Repressive histone marks, such as H3K9me1, H3K9me2, H3K9me3, H3K27me2 and H3K27me3 are largely over-mutated in comparison with active histone marks, such as H3K4me1, H3K4me2, H3K79me1,H3K79me2,H3K79me3, and H4K20me1 (P values range from 0.3482 to 2.429e-13 and are less than 0.05 in 95.83 % of cases for cancer somatic mutations, P values range from 0.8618 to 3.5742e-09 and are less than 0.05 in 73.33 % of cases for SNPs, Wilcoxon rank sum test). Furthermore, in order to further characterize the relation between somatic mutation, SNP rates and each feature, we constructed 2856 1-Mb windows, in which each row (1-Mb window) contains somatic mutation, SNP densities and 54 feature vectors (see “Methods” section). Correlation analyses were conducted between cancer somatic mutation, SNP densities and each feature vector. Features such as promoter, replication time, CDS, UTR are most negatively correlated with both somatic mutation and SNP densities (r = −0.3036 to −0.6178, P value <1.5233e-61 for somatic mutations; r = −0.0264 to −0.1219, P value = 1.6048e-01–7.2937e-11 for SNPs). Repressive histone marks, such as H3K9me1, H3K9me2, H3K9me3, H4K20me3, H3K27me2 show high positive correlations with both somatic mutation and SNP densities (r = 0.1336–0.6044, P value <1.1440e-12 for somatic mutations; r = 0.3393–0.5178, P value = 0 for SNPs) (Fig. 2). In general, SNP rates exhibit a large difference with somatic mutations, such as conserved regions and cTFBS (conserved transcription factor binding sites). These two regions are over-mutated in somatic mutations but protected from SNPs (Fig. 1). Recombination rates show strong positive correlation with SNPs but a relatively weak correlation with somatic mutations (r = −0.1210–0.0499, P value <7.8871e-03 for somatic mutations; r = 0.5015, P value = 0 for SNPs). Moreover, multiple features have contrasting correlations with somatic mutation and SNP rates, such as H3K4ac, H4K5ac, H3K4me1, H3K4me2, H4K20me1 and ncExon (Fig. 2), suggesting distinct mutation patterns of somatic mutations and SNPs in cancer genome.

**Fig. 1:** Densities of cancer somatic mutations of ccRCC associated to a wide range of genomic features chromosome by chromosome. For each chromosome, the size of each feature was calculated and numbers of somatic mutations were counted, somatic mutation densities were computed. The *red* and *blue dashed lines* stand for CDS and genome-wide average mutation densities. *CDS* coding sequence, *CR* conserved region, *ECS* evolutionarily conserved structure, *GCH* and *GCL* 1 Kb-windows with high and low GC content, *Exon.P* and *Exon.L*, *Intron.P* and *Intron.P* exon and intron of protein coding gene and lncRNA respectively, *PCgene* protein coding gene, *cTFBS* conserved TFBS, *UTR* Untranslated region, *PCgene.ER* and *PCgene.LR*, *LncRNA.ER* and *LncRNA.LR* early and late replicated protein coding gene and lncRNA, *PCgene.HE* and *PCgene.LE*, *LncRNA.HE* and *LncRNA.LE* high and low expressed protein coding gene and lncRNA, *RRH* and *RRL* 1 Kb-windows with high and low recombination rate, H3K4me1, H3K9ac, *etc*. histone methylation and acetylation data, *ncExon* non coding Exon

**Fig. 2:** Correlation coefficients of cancer somatic mutation (CSM), SNP densities with diverse genetic and epigenetic features at 1-Mb resolution

### Cancer somatic mutation (CSM) and SNP random forest models

Given the sparse number of cancer mutations, we built two random forest models, referred to as the CSM and SNP models, with 2856 1-Mb windows constructed above in order to analyze mutation distribution in more detail. %IncMSE is computed from permuting a predictor’s values over the original dataset, if a predictor is important in the model, the prediction error on the out-of-bag portion of the data (MSE for regression) will be increased [15]. We used %IncMSE to measure feature importance in the random Forest. In the CSM model, repressive histone marks such as H3K9me1, H3K9me2, H3K27me3, H3K27me2 and H4K20me3, replication time and promoter are among the most informative factors, which corresponds to the findings in the correlation analyses (Fig. 3a; Additional file 1: Figure S5). However, features such as CDS, UTR have medium importance in the CSM model, a possible explanation is these regions are relatively small in the genome and have little impact on genome-wide mutation rates, supporting that repressive histone marks, replication time and promoter contribute most to the CSM models. In the SNP model, the most important features are recombination rate, H4R3me2, H4K20me3, ECS, H3R3me2 and H3K27me2, which is in line with the correlation analyses above (Fig. 3b).

**Fig. 3:** Importance measured by %IncMSE for each feature in the CSM and SNP RF models **a** %IncMSE importance of all features in the CSM RF model; **b**  %IncMSE importance of all features in the SNP RF model

### Functionality and mutation frequency

Next, we asked whether mutation frequencies are associated to functionality and distribution of functional mutations. In order to examine this hypothesis, firstly, we constructed annotation data which are overlapping 1-Mb windows with a step size 1 Kb using all 54 features, CSM and SNP densities (CSM and SNP scores) were predicted with the CSM and SNP random models for each 1 Mb-window and cancer type and averaged on a 1 Kb scale (see “Methods” section). We applied SIFT and Mutation Assessor to predict damaging coding mutations for all cancer types. In total, 10,572, 1208,1625, 2519, and 7745, 1924,3009,3579 mutations were predicted as deleterious by SIFT and Mutation Assessor in ccRCC, liver cancer, lung cancer and melanoma respectively. We found markedly higher densities of deleterious mutations in the low CSM and SNP scoring regions as compared with those in the high CSM and SNP scoring ones. Moreover, negative correlations of average CSM and SNP scores were observed with densities of damaging mutations (r = −0.6034 to −0.9060 for CSM scores, r = −0.4721 for SNP scores, p value <0.05 in all cases), suggesting strong enrichment of deleterious mutations in the low mutated regions (Fig. 4a, b; Additional file 1: Figure S6). On the other hand, we computed functional scores for all non-coding mutations with FunSeq 2 and GWAVA and analyzed their distributions with respect to mutation rates. We observed that hypomutated regions with low CSM and SNP scores have higher average FunSeq 2 and GWAVA scores than hypermutated ones. Take the 200 Mb intervals with the highest and lowest CSM and SNP scores as examples, the 200 Mb interval with the lowest average CSM score has higher average GWAVA and FunSeq 2 scores than that with highest CSM score (*P* value <2.2e-16 in all cases, Wilcoxon rank sum test); The differences of average GWAVA and FunSeq 2 scores are relatively weak between the 200 Mb intervals with lowest SNP score and highest SNP score (P value = 0.0090 for GWAVA, P value = 0.161 for FunSeq 2, Wilcoxon rank sum test) (Fig. 4c, d; Additional file 1: Figure S7). Furthermore, we took 100 Mb lowest and highest scoring CSM, SNP regions respectively and analyzed their distributions across various genetic features. As expected, functionally important regions, such as CDS, exons, UTR, splicing sites of protein coding genes and miRNAs, have 2–48-fold higher enrichment of low CSM and SNP scoring regions than high CSM and SNP scoring regions (*P* value <2.2e-16 for all cases, Chi squared test), however, nearly functionally neutral regions, such as lncRNAs and intron of lncRNAs are 1.5–2-fold more enriched with high CSM and SNP scoring regions relative to low CSM and SNP scoring ones (*P* value <2.2e-16 for all cases, Chi squared test). Strikingly, fractions of low CSM and SNP scoring regions are 7~ times higher than those of high CSM and SNP scoring regions in cancer-related miRNAs and genes (*P* value <2.2e-16 in all cases, Chi squared test) (Fig. 5a; Additional file 1: Figure S8). In addition, ccRCC driver genes, VHL, PBRM1, TCEB1, BAP1 and SETD2, are all located in the low scoring 1-Kb windows, their average CSM scores are 21.436, 20.7088, 25.043, 20.7625 and 20.3447 respectively, which are less than the average (25.0582) in ccRCC. Lastly, we obtained non-coding disease-causing variants from HGMD and ClinVar databases and analyzed their distributions with regards to mutation rates. Disease-associated variants have lower average SNP and CSM scores than random SNPs (*P* value <2.2e-16 in all cases, Wilcoxon rank sum test) (Fig. 5b; Additional file 1: Figure S9). Low CSM and SNP scoring regions have higher enrichment of disease-causing variants than high CSM and SNP scoring ones. Take the lowest and highest CSM and SNP scoring 200-Mb intervals as examples, the former has an 14–117 times higher average densities of disease-causing variants than the latter (*P* value <2.2e-16 in all cases, Chi squared test). Significant negative correlations were observed between average CSM and SNP scores and densities of disease-associated variants (r = −0.6593 to −0.7790 for CSM scores,−0.5718 for SNP scores, P values <0.05 in all cases) (Fig. 5c, d; Additional file 1: Figure S10). All these findings support the fact that mutation rate is an important indicator of function and an influential factor on the distribution of functional mutations in cancer genome.

**Fig. 4:** The impact of CSM and SNP scores on the distribution of deleterious coding variants and functional non-coding variants. **a** average CSM scores correlate negatively with densities of deleterious coding variants predicted by SIFT and Mutation Assessor on a 200 Mb scale; **b** average SNP scores correlate negatively with densities of deleterious coding variants predicted by SIFT and Mutation Assessor on a 200 Mb scale; **c** The distribution of FunSeq 2 and GWAVA scores for non-coding variants with regards to CSM scores; **d** The distribution of FunSeq 2 and GWAVA scores for non-coding variants with regards to SNP scores

**Fig. 5:** The impact of CSM and SNP scores on the distribution of disease-causing variants from the ClinVar and HGMD databases. **a** The average fraction of 100 Mb low CSM, SNP, high CSM and SNP scoring regions in various features; **b** The distribution of CSM and SNP scores for ClinVar, HGMD disease-causing variants and random SNPs, random SNPs are 1 % SNPs randomly chosen from 1000 human genomes project; **c** The correlation of average CSM scores with densities of disease-causing variants on a 200 Mb scale; **d** The correlation of average SNP scores with densities of ClinVar, and HGMD disease-causing variants on a 200 Mb scale

## Discussion

In this study, we have characterized the mutation spectrum in four cancer types and observed a wide range of genomic features that contribute to somatic mutation variations across cancer genome. The most influential features are replication time, transcription levels, repressive, active histone marks and regulatory elements. In line with many studies [4–6, 16], we found late replicated genes are more mutable as compared to early replicated ones, the mechanisms underlying this phenomenon might be explained in two ways. First of all, exhaustion of dNTP in the late stages of DNA replication might cause increase of single strand DNA regions which are more susceptible to mutagenesis [17, 18]; Secondly, mutation repair systems might erode in the late replicated genes, leading to lack of efficient repair of mutation lesions [4]. Another feature associated with elevated mutation rate is low expressed genes. High transcription might reduce number of mutations through transcription-coupled repair (TCR), which would repair more DNA lesions along with global genome repair (GGR) than GGR could operate alone in low transcribed regions [19]. TCR also in part accounts for mutation frequency variations among repressive, active histone marks, exons, CDS, UTR and introns. Regions, such as repressive condensed chromatin and introns, are subject to increased mutation rates, which could be due to more active TCR in highly transcribed open chromatin, CDS, UTR and exons. Regulatory elements like promoters show reduced local densities of somatic mutations, probably due to the integrity of nucleotide excision repair pathway consisting of global genome repair and TCR, which guarantees the efficient removal of mutation lesions [20]. Lastly, we found that recombination rates positively correlate with somatic mutation and SNP densities, which is in agreement with Lercher’s study [21] ⁠but contrasts with that obtained by Renjamin’s study [7]. In particular, recombination rates are a major influential factor on the SNP density, which is mostly attributed to mutagenesis of recombination rate and faulty repair of the double-strand breaks that initiate recombination [21]. Consistent with mutation pattern in cancers, we found that repressive histone marks, promoter and replication time contribute most to the CSM models, features like recombination rate and chromatin organizations are most important for the SNP model.

Next, we asked whether mutation rate variations are a byproduct of mutation repair systems or represent cancer mutation selection and function in cancer. Here we showed mutation frequencies are linked to the distribution of functional mutations in cancers. Low mutated regions tend to enrich functional mutations, including deleterious coding mutations, functional non-coding mutations and disease-causing mutations, suggesting their importance in the formation of functionalities of somatic mutations. Another evidence that further support this idea is low mutated regions possess strikingly higher enrichment of functional regions, such as CDS, exons, UTR, splicing sites of protein coding genes, cancer-related miRNAs and cancer driver genes as compared to high mutated regions, which explains why low mutated regions are prone to form functional mutations. Currently, many studies prefer to emphasize the importance of hypermutation in cancer initiation and development [8, 19], and hypermutation is an indicator of positive selection in cancer genes and multiple computational methods have been developed to detect them [6, 11, 22]. Our study show that hypomutated regions are mutation constraints and associated to functions in cancer genome, which should draw more attention and work in the future.

## Conclusions

Taken together, somatic mutation densities vary largely across cancer genome, replication time, transcription levels, chromatin modifications and regulatory elements are among the features which most affect local mutation rates. To a large extent, mutation frequency is an indication of function and influence on the distribution of functional mutations in cancer.

## Methods

### Mutation data

Somatic variants were generated by whole genome sequencing of paired cancer and normal tissues and obtained from three studies: 2,011,261 variants from 25 melanoma patients [13], 1,845,976 variants from 24 lung adenocarcinoma patients, and 881,136 variants from 88 liver cancer patients [6] and 71,424 variants from 14 paired ccRCC and normal samples [12].Variants described as “substitution” or “indel” were both collected and are referred to collectively as mutations in the text. Germ line mutation data including 38,248,779 SNPs (single nucleotide polymorphism) were obtained from the 1000 genomes project [14] ⁠ (http://www.1000genomes.org). Disease-associated variants data come from ClinVar (Version 2014/03/03, 55,689 variants) [23] and HGMD [24] (Version 2014/04/14, 166,768 variants) databases which are two common curations of variants related to human inherited diseases, coding variants were removed in this study, forming 6045 and 13,108 disease-implicated variants in the non-coding genome.

### Genome-wide data resources

Human genome annotation were obtained from Gencode V21, including protein coding genes, exons, introns, UTR, non-coding exons (ncExon) ect [25]. Evolutionarily conserved bases with phast Cons score greater than 117 were identified through alignment of 46 mammalian genomes with human [26]. Evolutionarily conserved structures (ECS) are RNA secondary structures predicted with a nouvel pipeline based on RNAz and SISSIz in Smith MA’ study [27]. Promoters generated by the Gerstein lab are regulatory regions 2.5 Kb from transcription start sites (TSS) [28]. Genome-wide mapping of histone acetylation and methylation data of CD4+ T cell line were produced by ChIP-seq in Wang’s [29] and Barski’s study [30] respectively, all coordinates conversion from hg18 assembly to hg19 was performed with the UCSC Lift Over program [26]. Conserved TFBS (conserved transcription factor binding sites, cTFBS) were generated through aligning mouse and rat genomes with human [31]. Replication time data were obtained from Hepg2, Imr90, K562 and Bg02 cell lines for liver cancer, lung cancer, ccRCC and melanoma respectively (http://genome.ucsc.edu/) ENCODE, ‘Repli-seq track’ [31]. Genome-wide replication timing was mapped to protein coding genes and lncRNAs, the (G1b + S1)/(S4 + G2) ratio, early-to-late ratio, was determined for each protein coding gene and lncRNA. Genes that have a ratio greater than 1 or less than 1 were defined as early or late replicated genes respectively. Recombination rates (RR) were obtained from International HapMap Project (http://hapmap.ncbi.nlm.nih.gov/) and averaged over successive 1-Kb windows in human genome [32]. 1-Kb windows that have an average RR above 4.0 were regarded as high RR regions (RRH), while low RR regions are 1-Kb windows with recombination rate less than 0.5 (RRL). GC content denotes the percentage of G or C nucleotides per 1-Kb window. 1-Kb windows that have greater than 50 % or less than 30 % GC coverage are considered as high (GCH) or low GC regions (GCL) respectively [26].

RNA-seq data in sra format generated by sequencing 6 Hek293T cell lines were downloaded from NCBI (GSE55572) [33] for expression analysis in ccRCC. Read alignment was conducted with TopHat2 release 2.0.13 [34]. As for other cancer types, RNA-seq data in bam format were acquired from Hepg2, A549 and Nhek cell lines for liver cancer, lung cancer and melanoma respectively [31]. Read coverage was determined with bedtools v2.22.1 for lncRNAs and protein coding genes [35]. The number of reads per Kilobase per million reads (RPKM) was computed and averaged from three cell samples for each protein coding gene and lncRNA. Genes whose RPKM >20 or <0.25 were defined as high and low expressed respectively.

Cancer micro RNAs are a manual curation of mammalian miRNAs that have been experimentally characterized and actively involved in various cancers [36]. Cancer census genes are 547 cancer-driving genes annotated in COSMIC v71 (catalogue of somatic mutations in cancer) [37].

### Construction of 1-Mb windows and correlation analyses

We used 1-Mb window strategy to construct 1-Mb windows for correlation analyses between SNP, cancer somatic mutation densities and genetic features as well as fitting Random forest models. Non-overlapping 1-Mb windows were formed across human genome, cancer mutations and SNPs were mapped into them and the number of somatic mutations and SNPs were counted for each 1-Mb window. Genome-wide replication timing was mapped into 1-Mb windows and the (G1b+S1)/(S4+G2) ratio was computed for each 1-Mb window. Read coverage was determined with bedtools v2.22.1 for each 1-Mb window, exons from Gencode V21 were intersected with 1-Mb windows and the length of exons was then calculated for each 1-Mb window. The number of reads per Kilobase per million reads (RPKM) was computed and averaged from three cell samples for each 1-Mb window. Recombination rates (RR) were averaged over successive 1-Mb windows in the human genome. Regarding other features, the number of bases covered by each feature was calculated for each 1-Mb window. As a number of 1-Mb windows are lack of coverage of features and mutation information, partial 1-Mb windows were discarded, including 1-Mb windows defined as telomere, centromere, stalk, pericentromere, 1-Mb windows which are all undefined bases. The whole chromosome Y was ruled out from this study too, due to its consistently low mutation rates caused by gender bias. In total, 224.3 Mb regions were abandoned in this study, forming 2856 1-Mb windows and 56 columns corresponding to cancer somatic mutation density, SNP density and 54 features ranging from conserved regions, promoters to histone modifications. Correlation analyses between SNP, cancer somatic mutation densities and each feature were performed in R.

### Random forest model

The SNP and cancer somatic mutation (CSM) random forest (RF) models were constructed with the R random Forest package [15]. In the RF models, we used 2856 1-Mb windows constructed above and cancer mutation density (CSM model), SNP density (SNP model) as response variables and 54 genomic features as predictor variables to build two RF models, CSM and SNP models. All predictor values were plus one and log scaled to reduce the great variation of vectors. The number of trees was set to 500, mtry was set to 20 for CSM model and 15 for SNP model, all other parameters were set to default values. Model calibration and validation were described in the Additional file 2.

For CSM and SNP score prediction, we used the same 1-Mb window strategy as in the model building, however, the 1 Mb-window was slided across the human genome with a step size of 1 Kb. 1 Mb windows overlapping telomere, centromere, stalk or pericentromere regions, 1 Mb windows which are all undefined bases and chromosome Y were removed from the annotation data, resulting in 2,832,687 row annotations. The CSM and SNP scores were predicted using the two RF models for each 1 Mb window and averaged on a 1-Kb window scale.

### Correlation analyses between CSM, SNP scores and deleterious coding mutations, GWAVA and FunSeq 2 non-coding scores, disease-causing variants

Coding mutations mainly came from two sources for ccRCC: whole genome sequencing of 14 paired ccRCC samples and exome sequencing of 325 paired ccRCC samples from TCGA [38]. The coding mutations of other cancer types were obtained from the same sources as described in the section of “Mutation data”. Their functional impacts were predicted by SIFT [39], and Mutation assessor [40] respectively, variants were regarded as deleterious based on the following criteria: SIFT score <0.05, and Mutation Assessor socre >1.9. 70,659 ccRCC, 881,130 liver cancer, 1,623,242 lung cancer and 2,011,261 melanoma non-coding variants were scored with FunSeq 2 [41] (http://funseq2.gersteinlab.org/) and GWAVA [42] (https://www.sanger.ac.uk/sanger/StatGen_Gwava) respectively, all the parameters were set to default. Deleterious coding mutations, non-coding variants with GWAVA and FunSeq 2 scores and disease-causing variants from HGMD and ClinVar databases were mapped into 1-Kb windows which have average CSM and SNP scores. 1-Kb windows were then sorted based on SNP and CSM scores and divided into non-overlapping 200-Mb intervals respectively. For each 200-Mb interval, the following values were computed, including the average densities of deleterious coding mutations, disease-causing variants, average GWAVA and FunSeq 2 scores, average CSM and SNP scores. Correlation analyses were conducted in R between densities of deleterious coding mutations, disease-causing variants and average CSM and SNP scores.

### Statistical analyses

Data were presented as mean, statistical differences between groups were computed with the Chi squared test (chisq.test) or Wilcoxon rank sum test (wilcox.test), correlation analysis (cor.test) was conducted in R, *P* < 0.05 was regarded statistically significant and the null hypothesis was rejected.

## Additional files

**Additional file 1.** Supplementary figures.

**Additional file 2.** Calibration and validation of random forest models.

## References

[1] Hudson TJ, Anderson W, Artez A, Barker AD, Bell C, Bernabé RR, Bhan MK, Calvo F, Eerola I, Gerhard DS, Guttmacher A, Guyer M, Hemsley FM, Jennings JL, Kerr D, Klatt P, Kolar P, Kusada J, Lane DP, Laplace F, Youyong L, Nettekoven G, Ozenberger B, Peterson J, Rao TS, Remacle J, Schafer AJ, Shibata T, Stratton MR, Vockley JG (2010). International network of cancer genome projects. Nature.

[2] Chin L, Andersen JN, Futreal PA (2011). Cancer genomics: from discovery science to personalized medicine. Nat Med.

[3] Drier Y, Lawrence MS, Carter SL, Stewart C, Gabriel SB, Lander ES, Meyerson M, Beroukhim R, Getz G (2013). Somatic rearrangements across cancer reveal classes of samples with distinct patterns of DNA breakage and rearrangement-induced hypermutability. Genome Res.

[4] Stamatoyannopoulos JA, Adzhubei I, Thurman RE, Kryukov GV, Mirkin SM, Sunyaev SR (2009). Human mutation rate associated with DNA replication timing. Nat Genet.

[5] Woo YH, Li W-H (1004). DNA replication timing and selection shape the landscape of nucleotide variation in cancer genomes. Nat Commun.

[6] Lawrence MS, Stojanov P, Polak P, Kryukov GV, Cibulskis K, Sivachenko A, Carter SL, Stewart C, Mermel CH, Roberts SA, Kiezun A, Hammerman PS, McKenna A, Drier Y, Zou L, Ramos AH, Pugh TJ, Stransky N, Helman E, Kim J, Sougnez C, Ambrogio L, Nickerson E, Shefler E, Cortés ML, Auclair D, Saksena G, Voet D, Noble M, DiCara D (2013). Mutational heterogeneity in cancer and the search for new cancer-associated genes. Nature.

[7] Schuster-Böckler B, Lehner B (2012). Chromatin organization is a major influence on regional mutation rates in human cancer cells. Nature.

[8] Fox EJ, Prindle MJ, Loeb LA (2013). Do mutator mutations fuel tumorigenesis?. Cancer Metastasis Rev.

[9] Burns MB, Temiz NA, Harris RS (2013). Evidence for APOBEC3B mutagenesis in multiple human cancers. Nat Genet.

[10] Hoang ML, Chen CH, Sidorenko VS, He J, Dickman KG, Yun BH, Moriya M, Niknafs N, Douville C, Karchin R, Turesky RJ, Pu YS, Vogelstein B, Papadopoulos N, Grollman AP, Kinzler KW, Rosenquist TA (2013). Mutational signature of aristolochic acid exposure as revealed by whole-exome sequencing NIH Public Access. Sci Transl Med.

[11] Dees ND, Zhang Q, Kandoth C, Wendl MC, Schierding W, Koboldt DC, Mooney TB, Callaway MB, Dooling D, Mardis ER, Wilson RK, Ding L (2012). MuSiC: identifying mutational significance in cancer genomes. Genome Res.

[12] Sato Y, Yoshizato T, Shiraishi Y, Maekawa S, Okuno Y, Kamura T, Shimamura T, Sato-Otsubo A, Nagae G, Suzuki H, Nagata Y, Yoshida K, Kon A, Suzuki Y, Chiba K, Tanaka H, Niida A, Fujimoto A, Tsunoda T, Morikawa T, Maeda D, Kume H, Sugano S, Fukayama M, Aburatani H, Sanada M, Miyano S, Homma Y, Ogawa S (2013). Integrated molecular analysis of clear-cell renal cell carcinoma. Nat Genet.

[13] Berger MF, Hodis E, Heffernan TP, Deribe YL, Lawrence MS, Protopopov A, Ivanova E, Watson IR, Nickerson E, Ghosh P, Zhang H, Zeid R, Ren X, Cibulskis K, Sivachenko AY, Wagle N, Sucker A, Sougnez C, Onofrio R, Ambrogio L, Auclair D, Fennell T, Carter SL, Drier Y, Stojanov P, Singer MA, Voet D, Jing R, Saksena G, Barretina J (2012). Melanoma genome sequencing reveals frequent PREX2 mutations. Nature.

[14] Clarke L, Zheng-Bradley X, Smith R, Kulesha E, Xiao C, Toneva I, Vaughan B, Preuss D, Leinonen R, Shumway M, Sherry S, Flicek P (2012). The 1000 Genomes Project: data management and community access. Nat Methods.

[15] Breiman L (2001). Random forests. Mach Learn.

[16] Liu L, De S, Michor F (2013). DNA replication timing and higher-order nuclear organization determine single-nucleotide substitution patterns in cancer genomes. Nat Commun.

[17] Mirkin EV, Mirkin SM (2007). Replication fork stalling at natural impediments. Microbiol Mol Biol Rev.

[18] Yang Y, Sterling J, Storici F, Resnick MA, Gordenin DA (2008). Hypermutability of damaged single-strand DNA formed at double-strand breaks and uncapped telomeres in yeast Saccharomyces cerevisiae. PLoS Genet.

[19] Roberts SA, Gordenin DA (2014). Hypermutation in human cancer genomes: footprints and mechanisms. Nat Rev Cancer.

[20] Polak P, Lawrence MS, Haugen E, Stoletzki N, Stojanov P, Thurman RE, Garraway LA, Mirkin S, Getz G, Stamatoyannopoulos JA, Sunyaev SR (2014). Reduced local mutation density in regulatory DNA of cancer genomes is linked to DNA repair. Nat Biotechnol.

[21] Lercher MJ, Hurst LD (2002). Human SNP variability and mutation rate are higher in regions of high recombination. Trends Genet.

[22] Lawrence MS, Stojanov P, Mermel CH, Robinson JT, Garraway LA, Golub TR, Meyerson M, Gabriel SB, Lander ES, Getz G (2014). Discovery and saturation analysis of cancer genes across 21 tumour types. Nature.

[23] Landrum MJ, Lee JM, Riley GR, Jang W, Rubinstein WS, Church DM, Maglott DR (2013). ClinVar: public archive of relationships among sequence variation and human phenotype. Nucleic Acids Res.

[24] Stenson PD, Mort M, Ball EV, Howells K, Phillips AD, Thomas NS, Cooper DN (2009). The Human Gene Mutation Database: 2008 update. Genome Med.

[25] Harrow J, Frankish A, Gonzalez JM, Tapanari E, Diekhans M, Kokocinski F, Aken BL, Barrell D, Zadissa A, Searle S, Barnes I, Bignell A, Boychenko V, Hunt T, Kay M, Mukherjee G, Rajan J, Despacio-Reyes G, Saunders G, Steward C, Harte R, Lin M, Howald C, Tanzer A, Derrien T, Chrast J, Walters N, Balasubramanian S, Pei B, Tress M (2012). GENCODE: the reference human genome annotation for the ENCODE project. Genome Res.

[26] Karolchik D, Barber GP, Casper J, Clawson H, Cline MS, Diekhans M, Dreszer TR, Fujita PA, Guruvadoo L, Haeussler M, Harte RA, Heitner S, Hinrichs AS, Learned K, Lee BT, Li CH, Raney BJ, Rhead B, Rosenbloom KR, Sloan CA, Speir ML, Zweig AS, Haussler D, Kuhn RM, Kent WJ (2014). The UCSC Genome Browser database: 2014 update. Nucleic Acids Res.

[27] Smith MA, Gesell T, Stadler PF, Mattick JS (2013). Widespread purifying selection on RNA structure in mammals. Nucleic Acids Res.

[28] Khurana E, Fu Y, Colonna V, Mu XJ, Kang HM, Lappalainen T, Sboner A, Lochovsky L, Chen J, Harmanci A, Das J, Abyzov A, Balasubramanian S, Beal K, Chakravarty D, Challis D, Chen Y, Clarke D, Clarke L, Cunningham F, Evani US, Flicek P, Fragoza R, Garrison E, Gibbs R, Gümüs ZH, Herrero J, Kitabayashi N, Kong Y, Lage K (2013). Integrative annotation of variants from 1092 humans: application to cancer genomics. Science.

[29] Wang Z, Zang C, Rosenfeld JA, Schones DE, Barski A, Cuddapah S, Cui K, Roh T-Y, Peng W, Zhang MQ, Zhao K (2008). Combinatorial patterns of histone acetylations and methylations in the human genome. Nat Genet.

[30] Barski A, Cuddapah S, Cui K, Roh TY, Schones DE, Wang Z, Wei G, Chepelev I, Zhao K (2007). High-Resolution Profiling of Histone Methylations in the Human Genome. Cell.

[31] Rosenbloom KR, Sloan CA, Malladi VS, Dreszer TR, Learned K, Kirkup VM, Wong MC, Maddren M, Fang R, Heitner SG, Lee BT, Barber GP, Harte RA, Diekhans M, Long JC, Wilder SP, Zweig AS, Karolchik D, Kuhn RM, Haussler D, Kent WJ (2013). ENCODE Data in the UCSC Genome Browser: year 5 update. Nucleic Acids Res.

[32] Altshuler DM, Gibbs RA, Peltonen L, Altshuler DM, Gibbs RA, Peltonen L, Dermitzakis E, Schaffner SF, Yu F, Peltonen L, Dermitzakis E, Bonnen PE, Altshuler DM, Gibbs RA, de Bakker PIW, Deloukas P, Gabriel SB, Gwilliam R, Hunt S, Inouye M, Jia X, Palotie A, Parkin M, Whittaker P, Yu F, Chang K, Hawes A, Lewis LR, Ren Y, Wheeler D (2010). Integrating common and rare genetic variation in diverse human populations. Nature.

[33] Schwartz S, Mumbach MR, Jovanovic M, Wang T, Maciag K, Bushkin GG, Mertins P, Ter-Ovanesyan D, Habib N, Cacchiarelli D, Sanjana NE, Freinkman E, Pacold ME, Satija R, Mikkelsen TS, Hacohen N, Zhang F, Carr SA, Lander ES, Regev A (2014). Perturbation of m6A writers reveals two distinct classes of mRNA methylation at internal and 5′ sites. Cell Rep.

[34] Kim D, Pertea G, Trapnell C, Pimentel H, Kelley R, Salzberg SL (2013). TopHat2: accurate alignment of transcriptomes in the presence of insertions, deletions and gene fusions. Genome Biol.

[35] Quinlan AR, Hall IM (2010). BEDTools: a flexible suite of utilities for comparing genomic features. Bioinformatics.

[36] Xie B, Ding Q, Han H, Wu D (2013). MiRCancer: a microRNA-cancer association database constructed by text mining on literature. Bioinformatics.

[37] Forbes SA, Bindal N, Bamford S, Cole C, Kok CY, Beare D, Jia M, Shepherd R, Leung K, Menzies A, Teague JW, Campbell PJ, Stratton MR, Futreal PA (2011). COSMIC: mining complete cancer genomes in the catalogue of somatic mutations in cancer. Nucleic Acids Res.

[38] Chang K, Creighton CJ, Davis C, Donehower L, Drummond J, Wheeler D, Ally A, Balasundaram M, Birol I, Butterfield YSN, Chu A, Chuah E, Chun H-JE, Dhalla N, Guin R, Hirst M, Hirst C, Holt RA, Jones SJM, Lee D, Li HI, Marra MA, Mayo M, Moore RA, Mungall AJ, Robertson AG, Schein JE, Sipahimalani P, Tam A, Thiessen N (2013). The Cancer Genome Atlas Pan-Cancer analysis project. Nat Genet.

[39] Ng PC, Henikoff S (2003). SIFT: predicting amino acid changes that affect protein function. Nucleic Acids Res.

[40] Reva B, Antipin Y, Sander C (2011). Predicting the functional impact of protein mutations: application to cancer genomics. Nucleic Acids Res.

[41] Fu Y, Liu Z, Lou S, Bedford J, Mu XJ, Yip KY, Khurana E, Gerstein M (2014). FunSeq2: a framework for prioritizing noncoding regulatory variants in cancer. Genome Biol.

[42] Ritchie GRS, Dunham I, Zeggini E, Flicek P (2014). Functional annotation of noncoding sequence variants. Nat Methods.

